The article "Potential of solid dispersions to enhance solubility, bioavailability, and therapeutic efficacy of poorly water-soluble drugs: newer formulation techniques, current marketed scenario and patents" was retracted in 2022. Reason: plagiarism.

# Potential of solid dispersions to enhance solubility, bioavailability, and therapeutic efficacy of poorly water-soluble drugs: newer formulation techniques, current marketed scenario and patents

**DOI:** 10.1080/10717544.2020.1846638

**Published:** 2020-11-18

**Authors:** Sultan Alshehri, Syed Sarim Imam, Afzal Hussain, Mohammad A. Altamimi, Nabil K. Alruwaili, Fahad Alotaibi, Abdullah Alanazi, Faiyaz Shakeel

**Affiliations:** a Department of Pharmaceutics, College of Pharmacy, King Saud University, Riyadh, Saudi Arabia;; b College of Pharmacy, Almaarefa University, Riyadh, Saudi Arabia;; c Department of Pharmaceutics, College of Pharmacy, Jouf University, Sakaka, Saudi Arabia;; d General Directorate Health Affairs, Ministry of Health, Riyadh, Saudi Arabia

**Keywords:** Bioavailability;, marketed formulations;, dissolution;, solid dispersion;, patent status

## Abstract

In the last few decades, solid dispersion (SD) technology had been studied as an approach to produce an amorphous carrier to enhance the solubility, dissolution rate, and bioavailability of poorly water-soluble drugs. The use of suitable carrier and methodology in the preparation of SDs play a significant role in the biological behavior of the SDs. SDs have been prepared using a variety of pharmaceutically acceptable polymers utilizing various novel technologies. In the recent years, much attention has been paid toward the use of novel carriers and methodologies in exploring novel types of SDs to enhance therapeutic efficacy and bioavailability. The use of novel carriers and methodologies would be very beneficial for formulation scientists to develop some SDs-based formulations for their commercial use and clinical applications. In the present review, current literature of novel methodologies for SD preparation to enhance the dissolution rate, solubility, therapeutic efficacy, and bioavailability of poorly water-soluble drugs has been summarized and analyzed. Further, the current status of SDs, patent status, and future prospects have also been discussed.

## 1. Introduction

The paradigm of solubility challenges faced by formulation scientists is still largely unchanged. The poor aqueous solubility and subsequent dissolution rate of any drug are one of the most considerable challenges during formulation design and development. For the last two decades, the drug discovery and selection of new chemical entity (NCE) have taken a comprehensive scrutiny process through the use of combinatorial screening tools such as combination high throughput screening (Lipinski et al., 2001; Baird & Taylor, 2012). The drug molecules are classified as per the biopharmaceutics classification system (BCS), wherein a drug is considered as poorly aqueous soluble when the highest dose strength is not completely soluble in 250 mL aqueous media over the pH ranges of 1–8 at 37 °C (Vo et al., 2013). Nowadays, the pharmaceutical industry is facing major challenges to apply approaches that enhance the solubility and dissolution of poorly soluble drugs to get desired therapeutic effects (Kawabata et al., 2011). Various formulation approaches have been adopted to overcome the poor aqueous solubility problem (Vo et al., 2013). The solubility problem forced the pharmaceutical industry to search for different approaches to enhance drug solubility using the chemical, physical, and carrier-based approaches (Vasconcelos et al., 2007). The chemical method involves the molecular modification of drug structure resulting in the formation of new chemical salts or additive conjugate with varied pharmacokinetic and pharmacodynamics profiles (Seo et al., 2015). The physical method works by the principle of decreasing the size and increasing the contact surface area which leads to enhance solubility (Serrano et al., 2015). The different formulations approaches used to enhance the solubility are the production of lipid vehicles and/or surfactants based liquid systems (Gupta et al., 2013; Vasconcelos et al., 2016), or carrier-based solid formulations (Serrano et al., 2015). The solid dispersions (SDs) depict one of the most interesting approaches since it presents a reduced particle size, improved wettability and solubility, high porosity, and enhanced drug stability (Ohara et al., 2005; Vasconcelos et al., 2007). SD technique is the most widely accepted and successful strategy to enhance the solubility and release of poorly water-soluble drugs. The term SD has been defined as a dispersion of one or more active moiety in a suitable inert carrier or matrix in a solid-state. It can be prepared by different formulation methodologies (Paudwal et al., 2019). The drug molecule can be dispersed in a different form to prepare the SDs. It may be added as separate molecules, crystalline form, amorphous form in the amorphous or crystalline carrier. There are various well-established reported studies with gained advantages in solubility and dissolution rate enhancement. The advantages like reduced particle size possibly up to molecular level, enhanced porosity, wettability, and also the conversion of crystalline state particles into the amorphous state (Van den Mooter, 2011; Patel et al., 2015; Vasconcelos et al., 2016). Nowadays, there are number of marketed SDs have firmly established using different techniques for the formulation of poorly soluble drugs (Table 1). The main reason for the limited use of this technology is their physical instability during manufacturing and storage. The details of the marketed products have been given in orange book of USFDA. In the year 1985, first nabilone SD pharmaceutical product was approved by the FDA for the treatment of cancer. The most of the available marketed SD formulations have used cellulose polymers and povidones as the carriers. Hydroxyl propyl methylcellulose (HPMC) has been reported to act as a stabilizer by inhibiting the recrystallization of itraconazole (Sporanox^®^ oral capsule) and the supersaturated solution is kept stable for absorption from the intestine. Moreover, the phase separation can be mitigated by maintaining low molecular mobility of the matrix and drug during SD manufacturing process. The molecular mobility of the amorphous system depends on the composition and manufacturing process (Bhugra et al., 2007). Solid dispersions exhibiting high conformational entropy and low molecular mobility lead to form more physically stable SDs (Zhou et al., 2007). The molecular mobility can be decreased by using the polymers which can enhance the physical stability of amorphous drugs in SDs by increasing the *T*_g_ of the miscible mixture. The molecular mobility also decreased at normal storage temperatures, or by interacting specifically with drug functional groups (Taylor & Zografi, 1997; Vasconcelos et al., 2007). There are a series of considerable factors required to fabricate a successful product for commercialization. These points are taken into account to generate a proof of concept based on the evaluation parameters and manufacturing variable process. However, the technique has certain inherent limitation due to its translation to industrial scale-up, reproducibility of physicochemical properties on benchtop assessment, phase separation due to temperature-dependent stability (humidity and thermal mediated drug deterioration), and chances of drug crystallization during long term storage (Pokharkar et al., 2006; Vo et al., 2013). Phase separation and drug instability are the most common issues in the SD technique which might be prudent to correlate with incompatibility between drug and solvent and drug recrystallization from supersaturation solution. Such incompatibility arises owing to a significant difference in polarity and temperature-dependent supersaturated solubilization. The commercial products like Rezulin^®^, Isoptin SR^®^, Incivek^®^, and Norvir^®^ (Abbott Laboratory, Chicago, IL) were withdrawn from the market. It is evident for its withdrawal from the market due to recrystallization (changed in crystallinity resulted into reduced dissolution rate) of the drug from supersaturation solution on ageing. A thorough understanding of physicochemical features of drug, solvent, and matrix play a prime role to avoid possible chances of challenges. The sequential steps for formulation development of SDs are summarized in Table 2. There are many physicochemical parameters that may affect the SDs preparation. The factors like micromeritic property, specific surface area, pore volume, carrier molecular weight, carrier nature (crystalline, semi-crystalline, amorphous), carrier content, and carrier hygroscopicity are considered in SDs formulation. These parameters greatly affect the drug solubility, stability, and dissolution (Duong & den Mooter, 2016). The other physicochemical characteristics of carriers also considered the preparation of SDs and are summarized in Table 3. The objective of this review was to summarize and analyze various novel technologies of SDs preparation used for the enhancement of solubility, dissolution rate, therapeutic efficacy, and bioavailability of poorly water-soluble drugs. The current scenario, patent status, and future perspective of SDs have also been taken into consideration.

**Table 1.** Marketed solid dispersion formulations.

S. no.	Drug	Class	Method	Carrier	Manufacturer	Trade name	Dosage form	Year approval	USFDA orange book application number	Status
1	Nabilone	Anti cancer	Solvent evaporation	PVP	Valeant	Cesamet^®^	Capsule	FDA (1985)	N018677	Prescription
2	Itraconazole	Anti fungal	Fluid bed bead layering	HPMC	Janssen Pharmaceuticals Inc.	Sporanox^®^	Capsule	FDA (1992)	N020083	Prescription
3	Tacrolimus	Organ transplantation	Kneading, drying	HPMC	Astellas	Prograf	Capsules	FDA/MHRA (1994)	N050708	Prescription
4	Verapamil	Anti hypertensive	Hot melt extrusion	HPMC/HPC	Abbot	Isoptin SR	Tablets	FDA (1987)	N018593	Withdrawn
5	Troglitazone	Anti diabetic	Hot melt extrusion	HPMC	Pfizer	Rezulin^®^	Tablets	FDA (1997)	N020720	Withdrawn
6	Rosuvastatin	Anti hyperlipidemic	Spray drying	HPMC	Astra Zeneca	Crestor^®^	Tablets	2002 (FDA) 2004 (EMA)	N021366	Prescription
7	Duloxetine	Depression	NA	HPMCAS	Eli Lilly	Cymbalta	Capsule	FDA (2004)	N021427	Prescription
8	Lopinavir/Ritonavir	AIDS	Melt extrusion	PVP	Abb Vie	Kaletra	Tablets	EMA (2001) FDA (2005)	N021906	Prescription
9	Vildagliptin/Metformin HCl	Anti diabetic	Melt extrusion	HPC	Novartis	Eucreas/Galvusmet	Tablets	EMA (2007)	NA	NA
10	Fenofibrate	Hyperlipidemia	Spray melt	PEG6000 Poloxamer 188	Santorus Veloxis	Fenoglide	Tablets	FDA (2010)	N022118	Prescription
11	Etravirine	AIDS	HME	HPMC	J & J	Intelence	Tablets	FDA/EMA (2008)	N022187	Prescription
12	Tolvaptan	Hyponatremia	Granulation	NA	Otsuka	Samsca	Tablets	FDA/EMA (2009)	N022275	Prescription
13	Itraconazole	Onychomycosis	Hot melt extrusion	HPMC	Merz	Onmel	Tablets	FDA (2010)	N022484	Prescription
14	Everolimus	Organ transplantation	Co-precipitation	HPMC	Novartis	Certican/Zortress	Tablets	FDA/EMA (2010)	N021560	Prescription
15	Ritonavir	AIDS	HME	PVP	Abbvie	Norvir	Tablets	EMA(2009) FDA (2010)	N022417	Prescription
16	Vemurafenib	Cancer	Co-precipitation	HPMCAS	Roche	Zelboraf	Tablets	FDA (2011) EMA (2012)	N202429	Prescription
17	Telaprevir	Hepatitis	Spray drying	HPMCAS	Vertex	Incivek	Tablets	EMA/FDA (2011)	N201917	Withdrawn
18	Itraconazole	Fungal infection	Spray drying	HPMCP	Mayne	Lozanoc	Capsules	NA	NA	NA
19	Ivacaftor	Cystic fibrosis	Spray drying	HPMC-AS	Vertex	Kalydeco	Tablet	EMA/FDA (2012)	N203188	Prescription
20	Tacrolimus	Organ transplantation	Wet granulation	HPMC	Astellas	Advagraf/Astagraf XL	Capsules	FDA 2012	N204096	Prescription
21	Posaconazole	Fungal infection	HME	HPMCAS	Merck	Noxafil	Tablet	FDA (2013) EMA (2014)	N205053	Prescription
22	Etravirine	AIDS	Spray drying	HPMC	Tibotec	Intelence	Tablet	FDA 2008	N022187	Prescription
23	Regorafenib	Cancer	NA	Povidone K25	Bayer	Stivarga	Tablet	FDA 2012	N203085	Prescription
24	Silibinin	NA	Spray drying	Lecithin	Tianjin Tasly	Shuilinjia	Capsule	NA	NA	NA
25	Everolimus	Immunosuppressant	Spray drying	HPMC	Novartis	Votubia	Tablet	EMA/FDA (2010)	NA	NA
26	Nilvadipine	Hypertension	Spray drying	HPMC	Fujisawa	Nivadil	Tablet	NA	NA	NA
27	Griseofulvin	Fungal infection	Melt extrusion	PEG6000	Pedinol	Gris-PEG	Tablet	1982	N050475	Prescription
28	Florfenicol		NA	Enteric cellulose	Hebei Huaqiang	Flofenicol	Powder	NA	NA	NA
29	Ivacaftor; Lumacaftor	Cystic fibrosis	Spray drying	HPMCAS/SLS	Vertex Pharmaceuticals Inc.	Orkambi	Tablet	2015	N206038	Prescription

**Table 2.** The sequential steps of formulation development of SDs (Bedos et al., 2015; Beyerinck et al., 2015).

Steps	Criteria of selection
Selection of drug/carrier	Drug – crystalline, amorphous, metastable and should be compatible Carrier – crystalline, amorphous and should be soluble in common solvent Low melting point and high Tg Good compressibility index Solvent – capable of dissolving drug/carrier.
Literature report	Literature review and pharmacoeconomics Scale up and controlled process variables Intellectual property rights and patentability outcomes.
Method selection	Selection of suitable drug Screening of excipients and process variables Selection of method of preparation Control over challenges on final products (phase separation, precipitation, rubbery phase, drug degradation) Expected preclinical and clinical outcomes.
Proof of concept	Characterization Degree of crystallinity (XRD) Molecular interaction between drug and carrier (FTIR, DSC, NMR, IR). Dissolution study Transition temperature and enthalpy energy (DSC) Particle size analysis Surface morphology Stability study – humidity study, saturated solubility study
*In vitro in vivo* correlation and abbreviated new drug application.	Preclinical study in animal models to evaluate pharmacokinetic and toxicity study. Clinical study in human trials. Filling for approval before commercialization.

**Table 3.** Selection factors (physicochemical characteristics) of excipients for the development of solid dispersion (9110).

Details of excipients for the development of solid dispersion					
Commonly used solid carriers	Nature of solid carrier	Commonly used solvent	Melting point (°C)	Boiling point (°C) (vapor pressure at 25 °C)	Remark
Citric acid, tartaric acid, succinic acid, phosphoric acid	Acidic	Water	0	100 (3.16 kPa)	Water soluble solid carriers are suitable for melt method
Sodium acetate, sodium-o-hydroxy benzoate, sodium-p-hydroxy benzoate, sodium citrate, resorcinol, ascorbic acid	Hydrotropes	Methanol	–93.3	65 (16.9 kPa)	Volatile solvent suitable for thermolabile drugs
Dextrose, sorbitol, mannose, sucrose, maltose, galactose, xylitol, lactose, soluble starch, d-glucose, chitosan, galactomannan, amylodextrin, British gum	Sugars	Ethanol	–117	78.5 (5.79 kPa)	Volatile solvent suitable for thermolabile drugs
Gelucire 44/14, Poloxamer F-127, deoxycholic acid, Pluronic F68, Myrj 52, sodium lauryl sulfate, Tween 80, Span 80, vitamin E TPGS, docusate sodium, polyoxyethylene stearate	Surfactants	Ethanol	–117	78.5 (5.79 kPa)	Gelucire and TPGS commonly used
PEG-4000, PEG 6000, polyvinyl pyrrolidone (PVP), β-cyclodextrin, hydroxypropyl-β-cyclodextrin, Eudragit L100 sodium salt, sodium salt of crystalline microcellulose, hydroxy propyl methyl cellulose, methyl cellulose, guar gum, xanthan gum, dextrin	Polymers	Isopropyl alcohol	–127	82.4 (5.85 kPa)	Tackiness observed due to PEG and PVP
Dicalcium phosphate, silica gel, hydroxy alkyl xanthene, urethane, urea, skimmed milk, pentaerythritol	Others	Chloroform	–63	62 (26.1 kPa)	Volatile solvent suitable for thermolabile drugs

## 2. Classification of SDs

It is broadly classified on the basis of carrier used to prepare the SDs. The used carriers determine the final formulation properties and can be categorized into first, second, third, and fourth generation.

### 2.1. First generation

In this type, SDs are comprised of the crystalline carrier (urea, sorbitol, and mannitol) and crystalline drug (Sekiguchi & Obi, 1961; Vo et al., 2013). The urea-based SD exhibits high solubility in water and organic solvents, but the sugar-based SDs have poor solubility in an organic solvent and also the high melting point. Therefore, sugar has been avoided as a carrier to prepare SDs prepared by melting method. In the case of crystalline SDs, the crystalline carrier used to prepare a eutectic mixture or monotectic mixture. The crystalline state drug dispersed to the crystalline carrier. The solubility and dissolution of drug-enhanced by reducing the particle size, wettability, and alteration in the polymorphic state. The main drawbacks of crystalline SDs are the high carrier thermodynamic stability lead to decrease in the dissolution rate in comparison to amorphous SDs (Sekiguchi & Obi, 1961). The first formulation was reported by Sekiguchi & Obi (1961) and they used urea as a carrier to formulate sulfathiazole eutectic mixture (Sekiguchi & Obi, 1961). The prepared formulation reported the significantly enhanced dissolution in comparison to the physical mixture. The SD prepared with sugar-based carriers mainly lead to increase in surface area of drug to carrier, enhance wettability, and consequently solubility (Das et al., 2011). In other research, Okonogi et al. prepared ofloxacin-SD using the carrier urea and mannitol (Okonogi et al., 1997). They reported the enhanced dissolution and solubility than mannitol based SD. Among these two carriers, urea-based SD showed a more pronounced effect than mannitol-based SD. The higher solubility was also achieved due to the greater reduction in the crystallinity by the urea based SDs (Okonogi et al., 1997). The dissolution of clotrimazole was enhanced by SD using the carriers like d-mannitol, d-fructose, d-dextrose, and d-maltose. The SDs were prepared by fusion method by taking the different drug carrier ratio. The formulation showed many times enhancement in solubility in comparison to a conventional drug suspension. The dissolution study results revealed improved release behavior at 1:3 drug mannitol ratio (Madgulkar et al., 2016).

### 2.2. Second generation

The second-generation SD is comprised of amorphous carriers which are mainly polymers (synthetic polymers and natural polymers). The selection of carrier/matrix is a very important and critical step in the formulation of SDs. Based on the physical state of drug, the second generation SDs further classified into amorphous solid solution and amorphous solid suspensions (Karagianni et al., 2018). In amorphous solid solution, the drug and amorphous carrier are completely miscible to form molecularly homogenous mixture while amorphous solid suspension consists of two separate phases. In this type of systems, the drug particles are in the amorphous state and dispersed in the amorphous carrier. The presence of an amorphous carrier in SD helps to increase the wettability and dispersibility of the drug. It also helps to reduce the precipitation of drug when SDs dissolved in the aqueous phase (Crowley et al., 2007; Chauhan et al., 2013). The high dissolution can be achieved due to the low thermodynamic stability of the used carrier. There are a large number of natural and synthetic polymers used in this type of SDs. The polymers like povidone, polyethylene glycols (PEGs), hydroxypropylmethyl cellulose (HPMC), hydroxypropyl cellulose (HEC), and starch can be used to prepare these SDs. These polymers are soluble in an organic solvent or an aqueous solvent. Therefore, these polymers can be used to prepare the SDs by the solvent evaporation method. The polymers like polyvinyl pyrrolidone (PVP) and PEG-carrier-based felodipine SDs were prepared and evaluated by Karavas et al. (2007). Fourier transform infrared (FTIR) study revealed that in felodipine–PVP SDs, the drug was found in amorphous form but in case of PEG-carrier based SD, the drug was found in crystalline form. There was greater hydrogen boding observed with PVP carrier than PEG carrier (Ganesan et al., 2015). In another research work, hydrochlorothiazide loaded SDs were prepared using ethyl cellulose (EC) and HPMC carriers. The result of the study depicted a significantly enhanced dissolution profile (Ganesan et al., 2015). The amorphous fenofibrate (FB) SDs were prepared using the carriers HPMC-E5, HPMCP-55, HPMC-AS, and Soluplus. The dissolution study results revealed improvement in the release profile. The release profile followed the following order FB-HPMC-E5 > FB-HPMC-AS. Further, the prepared formulation evaluated for the pharmacokinetic study and results revealed significant enhancement in bioavailability. This result was achieved by the complete dissolution of FB in the proximal small intestine (Zhang et al., 2012). The solvent evaporation method was used to prepare diclofenac sodium SDs using Eudragit-E100 as the carrier. The prepared SDs were evaluated for solubility and the result revealed 0.823 mg/mL solubility of diclofenac in SD whereas pure diclofenac sodium showed only 0.014 mg/mL solubility. There was an approximately 58.8-fold enhancement in solubility by SDs compared to the pure drug. The dissolution result showed SD release was approximately 60% at 1.2 pH in 2 h whereas, pure drug depicted less than 10% release at same time point due to small particle size and enhanced wettability (Jafari, 2013).

### 2.3. Third generation

The third generation SD is prepared with the addition of surface-active agents or self-emulsifiers along with carriers. There is a significant improvement in solubility and drug release rate achieved and the problems like precipitation and recrystallization can be overcome. These surfactants are used as process aids and additives and act as solubility enhancer for the supersaturated solution system. The physical and chemical stability can also be enhanced with the enhancement of dissolution. It acts by improving the drug wettability and also able to prevent drug precipitation. It absorbs to the outer surface of particles or forms micelle to encapsulate the drug. There are several surfactants like Poloxamer, Gelucire 44/14, Soluplus, sodium lauryl sulfate (SLS), Tween 80, and Compritol were commonly used to prepare this type of SDs. Among these surfactants, Poloxamer is the most commonly used carrier and recently Soluplus has shown very significant result in the preparation of SDs by melt extrusion technology (Shah et al., 2013). The drugs like ibuprofen (IBU) and ketoprofen-loaded SDs were prepared using carriers like Poloxamer 407 and 188. The prepared samples were evaluated for the spectroscopy study and the results of the study revealed hydrogen bond formation between drug and carrier. The drug carrier ratio (2:1) revealed no crystal formation and conversion of the drug in amorphous form. There was significantly higher dissolution found with the formation of SDs (Ali et al., 2010). SLS-based sugar glass SDs were prepared and their results were compared with a standard tablet. The comparative dissolution study was performed and the results revealed marked enhancement in the dissolution. The presence of SLS as a carrier in the SDs prolonged the dissolution of. SLS helps to prolong the release and also help to maintain the high drug concentration in the near vicinity of the dissolving tablet during the dissolution process (De Waard et al., 2008).

Ketoconazole SD was prepared in different ratio by grinding method using Pluronic F127 as a carrier (Karolewicz et al., 2014). The prepared SDs were evaluated for different physicochemical parameters. The prepared samples showed that ketoconazole and Pluronic F127 form eutectic system of ketoconazole (containing ketoconazole 4.4% w/w) at the eutectic point. There was significantly enhanced dissolution was observed for ketoconazole with the addition of SLS (0.5% w/v). The enhancement in dissolution was achieved due to the increased solubilization of ketoconazole. In another study, lovastatin-loaded Pluronic F127 SD was prepared using kneading method (Karolewicz et al., 2016). The prepared SD was evaluated for dissolution profile in phosphate buffer at pH 7 with SLS (0.5%). The results of the study revealed 16.53% drug release by pure lovastatin in 24 h, whereas formulation containing lovastatin (50–80% w/w) released 100% release in 4 h. The same research group prepared FB SD by fusion method using Pluronic F127 as a carrier (Karolewicz et al., 2016). There was no interaction between drug and carrier which was observed by XRD, DSC, and FTIR study. The intrinsic dissolution study revealed 134-fold enhancement in dissolution for the sample containing the drug carrier ratio of 30:70% w/w. Karolewiczi et al. prepared acyclovir SD using Pluronic F127 and evaluated for different parameters (Karolewicz et al., 2016). The prepared SDs assessed for dissolution study and the results of study showed marked enhancement in dissolution with minimum amount of the carrier. In another study, the effect of Soluplus^®^ was assessed on the fluconazole-loaded SD (Nowak et al., 2019). The samples were prepared by different techniques like spray drying and fusion methods. The important findings of the study were the drug carrier ratio and method of preparation. The spray-dried sample showed slower drug release as compared to crystalline fluconazole. The slow drug release was found due to the slow diffusion of the drug molecules from thick polymer gel formed over the particles. In addition, the sample having the drug carrier ratio (10:90) stayed stable in amorphous state for 14 days.

### 2.4. Fourth generation

The poorly water insoluble drugs having short biological half-life can be used to prepare fourth generation SDs. It is called as controlled release SD (CRSDs). The two main targets can be achieved by preparing CRSDs like enhancement of drug solubility and controlled drug release pattern. In this type of SD, the poorly water-soluble drugs molecularly dispersed in the carrier. It can deliver an optimum amount of drug for an extended period. There are wide range of advantages are reported for poorly water-soluble drugs (Desai et al., 2006). There are wide range of polymers like EC, Eudragit, Carbopol, and poly(ethylene oxide) (PEO) used to prepare this type of SDs. These types of polymers having the property of low solubility which can help to sustain the drug release. Water-soluble carriers improve the solubility and dissolution, while water insoluble carrier or swellable carriers (EC, PEO, and carboxyvinyl polymer) are used to prolonged the release in controlled manner in the dissolution medium. These polymers are either water insoluble or dissolve very slowly in water responsible for sustained release of poorly water-soluble drugs. The extended-release SD of indomethacin was prepared using EC and HPMC (1:1) as the carriers. The study reported a strong hydrophobic interaction between carrier and drug at low pH and lead to slow dissolution (Ohara et al., 2005). In another research, Cui et al. formulated nitrendipine-SD incorporated sustained-release microspheres. The formulation was prepared using HPMCP-55 and Aerosil as the carrier systems. The bioavailability study results revealed a prolonged drug absorption profile in comparison to the reference tablets (Baypress™) and the conventional tablets (Cui et al., 2003). Aceclofenac-loaded PEO-based SD was prepared and evaluated for dissolution profile. The results revealed enhanced dissolution of drug with the addition of surfactant compared to the pure drug. The formulation showed retarded drug release in a zero-order manner due to the water swellable property of PEO (Tran et al., 2010).

## 3. Processing techniques

There are different process techniques used to prepare amorphous SDs. These processes are used to prepare few to hundred grams of finished SDs formulations. Table 4 depicts some of the recent application of laboratory scale prepared SDs with their findings.

**Table 4.** Overview of recently published SDs prepared using novel techniques.

Drug	Carrier	Method	Inference	References
Nifedipine, efavirenz	Hydroxypropyl methylcellulose acetate succinate	Hot melt extrusion	The inhibitory effects depend on the hydrophobic interactions between drug and polymer, and the dissolution dose of the drug	Sarabu et al. (2020)
Mefenamic acid	EudragitVR EPO	Hot melt extrusion	Mefenamic acid SD showed significant rat palatability tastes as compared with pure and marketed MA	Alshehri et al. (2019)
Mefenamic acid	Kollidon^®^ 12 PF and 17 PF	Hot melt extrusion	The *in vitro* release study demonstrated an immediate release for 2 h with more than 80% drug release within 45 min in matrices containing MgO and PEG in combination with polyvinylpyrrolidone when compared to the binary mixture, physical mixture, and pure drug.	Alshehri et al. (2017)
Carbamazepine	Soluplus^®^	Hot melt extrusion	The hardness and sphericity of drug were optimized.	Alshetaili et al. (2016)
Piperine	Eudragit^®^ EPO, Kollidon^®^ VA 64, Soluplus^®^	Hot melt extrusion	The permeability studies demonstrated the enhancement in piperine absorption of 10% w/w piperine/Soluplus^®^ extrudates up to 158.9 μg/5 mL compared with pure piperine at 1.3 μg/5 mL within 20 min.	Ashour et al. (2016)
Lansoprazole	Kollidon^®^ 12 PF, Lutrol^®^ F 68, MgO	Hot melt extrusion	The drug release and stability of drug was enhanced using hot melt extrusion technology compared with pure drug.	Alsulays et al. (2017)
Aripiprazole	Kollidon^®^ 12 PF (PVP) and succinic acid	Hot-melt extrusion	The oral bioavailability (*C*_max_ and AUC_0–12_) of N6 was significantly improved when compared to the pure aripiprazole.	McFall et al. (2019)
Hydrocortisone	Polyethylene glycol 4000 (PEG 4000), Kolliphor^®^ P 407	Spray drying	The PEG 4000 appears to be controlling the release of hydrocortisone *in vivo* after oral administration	Altamimi et al. (2019)
Apigenin	Pluronic-F127	Microwave irradiation	The enhancement in oral bioavailability of APG from microwave SD (319.19%) was 3.19-fold as compared with marketed capsule (100.00%)	Alshehri et al. (2019)
Mefenamic acid and flufenamic acid	Pluronic F127^®^ (PL), Eudragit EPO^®^ (EPO), polyethylene glycol 4000 (PEG 4000), Gelucire 50/13 (GLU)	Microwave irradiation	The SDs of MA and FFA prepared using PEG 400 showed higher drug release profile in comparison with those prepared using PL, EPO, or GLU	Alshehri et al. (2017)
Nifedipine, sulfamethoxazole	Soluplus^®^, PEG 6000	Spray drying, lyophilization	The drug dissolution rates were significantly enhanced	Altamimi & Neau (2017)
Efavirenz	Soluplus^®^	Spray-drying	Solubility and dissolution rate of efavirenz was enhanced by spray-dried solid dispersions	Lavra et al. (2017)
Apigenin	Pluronic F 127	Spray drying	Significant increase in the dissolution rate and bioavailability of the spray dried apigenin SDs.	Altamimi et al. (2018)
Sirolimus	Eudragit^®^ E HPMC	Spray drying	Solid dispersion significantly improved oral absorption of sirolimus. E-SD significantly inhibited the degradation of sirolimus in a dose-dependent manner and the precipitation of sirolimus compared to hydroxypropylmethyl cellulose (HPMC).	Cho et al. (2015)

### 3.1. Cryogenic processing techniques

The cryogenic processing techniques have the advantage to prepare SDs of thermolabile drugs. These methods include spray freeze drying (SFD) and ultra-rapid freezing (URF). These methods of SD preparation work on the principle of increasing the freezing rate compared to the conventional freeze-drying technique. In both of these methods, the procedure is performed under sub-ambient conditions. There may be fewer chances of drug degradation due to no contact between heat or air that may promote drug degradation during the drying process. In the SFD technique, the reduction of particle size takes place without the application of intense frictional or mechanical forces which lead to the degradation of drug particle by thermal stress (Purvis et al., 2007). The drug and carrier solution are sprayed into the cold air dried container and the frozen droplets are further lyophilized using SFD technique. There may be fewer chances of phase separation due to the direct contact of drug particles with the cooling agents and fast vitrification. This method converts the drug particles in the amorphous state due to the fast freezing process and protects the molecular arrangement into a crystalline state (Tong et al., 2011). The URF involves the application of thermal conductivity between 10 and 20 W/(mK) with a solid cryogenic substrate (Vo et al., 2013). The cryogenic solid substrate is applied to a frozen drug–polymer sample and the particles are collected from the solvent by lyophilization (Overhoff et al., 2007). In this method, the supercooling is very fast and the nucleation of drug crystals is reduced or completely prevented, leading to the amorphous morphology after lyophilization (Vishali et al., 2019).

### 3.2. Freeze drying

The freeze-drying method is the alternative method to the solvent evaporation method. It is suitable for the thermolabile drugs because minimal thermal stress is applied. The method of preparation involves two steps, i.e. freezing and lyophilization. In this method, the lyophilized molecular dispersion is prepared by dissolving the drug and carrier in a suitable solvent. The samples are then frozen in a liquid nitrogen (Onoue et al., 2013). Initially, the API and carrier solution are kept in liquid nitrogen until it is fully frozen and then the frozen sample is lyophilized (van Drooge et al., 2006; Van Drooge et al., 2006). The main advantage of this technique is the low risk of phase separation. The SDs of nifedipine and sulfamethoxazole were prepared by freeze-drying method using Soluplus and PEG 6000 as the carriers. The prepared SDs were evaluated for the physicochemical and *in vitro* characteristics. The enhanced dissolution and stability of both drugs were found compared with pure drugs (Altamimi & Neau, 2017). In another study, an exemestane-loaded SDs were prepared using the phospholipid/sodium deoxycholate carriers. The prepared SDs were evaluated for the solubility and oral bioavailability. The results of the study revealed a significant enhancement in the solubility and dissolution from SDs in comparison to the pure drug. The bioavailability study results depicted a significant enhancement in bioavailability in comparison with pure drug. The pharmacokinetic parameters like area under curve (AUC) were found to be 2.3-fold higher than pure drug (Kaur et al., 2017). The applicability of this technique was further used to prepare flutamide SDs using the carriers PVP K30, PEG 6000, and Poloxamer 407. The prepared SDs were evaluated for dissolution study and SDs prepared with Poloxamer 407 showed maximum drug release as compared to SDs prepared with other carriers. The release pattern was found as PVPK30 > PEG6000 after 30 min study (Elgindy et al., 2011).

### 3.3. Fluid-bed coating

The fluid-bed coating technique is the another technique used to prepare SDs. In this method, the drug and carriers are first dissolved in a suitable solvent. Then, the prepared solution is sprayed through nozzle onto the surface (Sun et al., 2008; Zhang et al., 2009). The solvent is evaporated by the application of air and then the samples are co-precipitated simultaneously by depositing on the surface (Lu et al., 2009). The main advantage of this method is that the prepared SDs granules or pellets can be directly used to prepare tablets or encapsulate into capsules. The FB and silymarin SDs were prepared by fluid-bed coating technique and reported the enhanced bioavailability of both drugs (Sun et al., 2008).

### 3.4. Spray drying

This method (Figure 1) is one of the most common methods used to prepare SDs due to the advantage of good size uniformity, high recovery, and less cost in large scale production (Bikiaris, 2011; Smithey & Taylor, 2013). In this method, the rapid solvent evaporation takes place and quick conversion of a drug-carrier solution to solid drug-carrier particles takes place (Paudel et al., 2013). The drug-carrier solution or suspension droplet is transported to the nozzle entrance using a pump and the breakdown of large droplets into fine droplets takes place with the large specific surface area. The formation of SD takes place by the rapid evaporation of the solvent and the size of particles optimized by adjusting the droplet size via a nozzle. The spray drying prepared SD showed the particles in the amorphous state and lead to significantly enhanced solubility and dissolution rate. There are several works in literature which reported the use of spray drying technique to prepare the SDs (Pawar et al., 2016; Pradhan et al., 2016; Herbrink et al., 2017; Al-Zoubi et al., 2018). The drugs used to prepare SD for enhancing the solubility of poorly water-soluble drugs such as nilotinib (Herbrink et al., 2017), spironolactone (Al-Zoubi et al., 2018), valsartan (Pradhan et al., 2016), and artemether (Pawar et al., 2016). Nilotinib-loaded SD was prepared using Soluplus as a carrier. The *in vitro* drug release study results revealed drug:Soluplus (1:7) ratio showed significant enhancement in the drug solubility compared with pure drug. The enhancement was found to be of 630-fold in comparison with the pure drug (Herbrink et al., 2017). In another research study, artemether-Soluplus-SDs were prepared and evaluated for dissolution study. The result of the study revealed the optimal ratio of artemether:Soluplus was found to be 1:3. The optimized ratio releases about 82% drug in 1 h which was 4.1-fold higher than the pure drug (20%) (Pawar et al., 2016).

**Figure 1.** Schematic working diagram of spray dryer.

Our group studied the hydrocortisone (HCT) SDs to investigate the bioavailability on rat model using PEG 4000 and Kolliphor^®^ 407 as the carriers. The SDs were prepared using spray drying technique and evaluated for physical and chemical characterization. The comparative *in vitro* and *in vivo* studies were conducted to evaluate the dissolution and bioavailability. The prepared SDs showed elongated leaf-shaped particles structure and also the formation of new bonds was suggested due to the change in the vibrational wave numbers. Further, the significant improvement in the *in vivo* study was found in the spray-dried formulation over the neat HCT. There was a twofold enhancement in the AUC and MRT was exhibited for spray-dried HCT: PEG 4000 SD (Altamimi et al., 2019). The same research group prepared spray-dried apigenin SD using Pluronic F 127 as a carrier. The developed SDs were evaluated for different physicochemical characterization, dissolution study, and *in vivo* study. The results of *in vivo* study revealed around fivefold enhancement in *C*_max_ for spray-dried SDs compared with than non-spray dried materials. The prepared drug:polymer (1:4 ratio) formulation showed elongated particles, complete lack of crystallinity leads to a significant increase in the dissolution rate and bioavailability (Altamimi et al., 2018). The solubility and dissolution of efavirenz, a practically insoluble drug, belongs to BCS class II (low solubility/high permeability) was enhanced by preparing SDs using the water-soluble carrier Soluplus^®^. The formulations were prepared by the spray drying method. The solubility and dissolution results revealed a remarkable enhancement in the spray-dried solid formulations (Lavra et al., 2017). Another SDs formulation of sirolimus was designed using Eudragit^®^ E/HCl as a carrier to evaluate the solubility and bioavailability enhancement. The formulation was prepared by the spray drying process and evaluated for different parameters. The pharmacokinetic study results indicated that prepared SD significantly improved oral absorption of sirolimus (Cho et al., 2015).

### 3.5. Microwave irradiation

Microwave irradiation (MWI) is electromagnetic irradiation found between the infrared (IR) and radio frequencies in the range of 0.3–300 GHz. Most of the MW works at a frequency of 2.45 GHz (all domestic and industrial MW devices operate at a frequency of 2.45 GHz equivalent to 12.25 cm wavelength). The microwave can easily penetrate in any materials and at the same time allows the generation of heat at any point of the sample. The characterization can be done by the presence of dipole moment in the molecules which help to absorb the MW energy and transform it into heat (Mavandadi & Pilotti, 2006; Bikiaris, 2011). One of the most important MW applications is the enhancement of dissolution rate of poorly water-soluble drugs. The application of MWs in the preparation of SDs appears to present several desirable attributes. Apart from the improvement of drug dissolution, the lower thermal treatment, which corresponds to a reduced risk of decomposition of heat-sensitive drug substances, and the shorter preparation time, make MW application a promising alternative to conventional methods for the preparation of SDs. The first research report published using MW technique is the formulation of felodipine loaded SDs for the enhancement of dissolution. In this technique, the SDs prepared by heating the physical mixture (drug and carrier as silicon dioxide) in a microwave oven (Kerc et al., 1998). In another research, poorly water-soluble drug nimesulide SDs has been prepared using the carrier Gelucire 50/13, Poloxamer 188 as a surfactant. They reported the enhanced solubility and dissolution of the used drug (Moneghini et al., 2009). The used samples have been irradiated due to the application of MW and the crystalline sample converted to an amorphous state. The effect of the MW irradiation on the tested nimesulide SDs performed by the dissolution study for both carriers treated samples. The dissolution comparison has been done with the pure drug and physical mixture. There was a remarkable enhancement in drug release was achieved by the samples prepared by the MW method. The SDs sample prepared with Gelucire 50/13 (1:2 w/w) showed about 90% drug release in 13 minutes, whereas the physical mixture showed 74% drug release at the same time. The corresponding percentage for the pure drug was only 18%. MW was used to prepare fast release SDs or sustained-release SDs of IBU (drug characterized by a low melting point) with PVP/VA 60/40 and HP-β-CD (Moneghini et al., 2008).

Mefenamic acid and flufenamic acid (FFA) SDs were prepared and evaluated for the enhancement of solubility and dissolution rate. The SDs were prepared using the solvent-free MWI technique using the different carriers. The prepared MWI samples were characterized for physicochemical parameters and drug release profile. The prepared SDs revealed enhanced dissolution rate of both drugs using PEG 400 carrier as compared to other carriers. The selected SDs showed significant % inhibition in comparison with pure MA (68.09% after 4 h) and pure FFA (55.27% after 4 h) (Alshehri et al., 2017). In another study, the same researchers reported the effect of Pluronic F127 as a carrier with apigenin SDs prepared by different methods like MWI, melted, and kneaded techniques. The different SDs were prepared and evaluated for the physicochemical characterization, *in vitro* drug release/dissolution profile, and *in vivo* pharmacokinetic studies. The physicochemical evaluation results revealed the successful formation of apigenin SDs. The *in vitro* dissolution and *in vivo* pharmacokinetic results suggested a significant enhancement in the release, as well as oral absorption of apigenin from SD, prepared using MWI and melted techniques (Alshehri et al., 2019). Recently, Alshehri et al. prepared luteolin (LT)-loaded SD using PEG 4000 as a carrier. They used different methods like fusion, solvent evaporation, and MWI to prepare LT-SDs. The comparative dissolution study was performed and the results revealed the SD prepared by MWI technique depicted maximum drug release (i.e. 97.78 ± 4.41%) with the ratio of LT and PEG 4000 (1:2). The MWI SDs showed maximum drug release due to greater solubility of LT and lower particle size. The same samples also showed the significantly higher radical scavenging activity than pure LT (Alshehri et al., 2020).

### 3.6. Co-precipitation method

The co-precipitation method used to prepare SDs because it does not require an elevated temperature. The less volatile solvents used to prepare SD and can be easily washed with aqueous media to completely remove the organic solvents (Sertsou et al., 2002). The selection of suitable polymer, solvent, and anti-solvent system is important parameters to control the precipitation. The drug and polymer carrier are completely dissolved in an organic solvent and finally the addition of an anti-solvent in the above mixture which leads to precipitation of the drug and carrier. The formulated sample is filtered, washed to remove the residual solvents, and finally dried to get micro precipitated bulk powder. The polymers and organic solvents used to prepare the SD by this method are polyvinyl phthalate, polymethylacrylate, dimethylacetamide, and dimethyl formamine. These types of solvents used for this method due to their excellent solvency power for the high molecular weight polymers (Shah et al., 2012). Dong et al. prepared and evaluated BCS class II drug-loaded SDs using HPMC-AS as a carrier. The SDs were prepared using co-precipitation and hot melt extrusion (HME) methods to compare with each other. The prepared samples were evaluated using PXRD technique to evaluate the physical state of the drug. The results revealed that the drug was found in amorphous state in SDs (Dong et al., 2008).

### 3.7. Electrostatic spinning

This method of preparation is a combination of SDs and nanotechnology. The advantage of this method is the availability of extremely high surface area per unit mass of fibers which promotes the fast and efficient solvent evaporation (Yu et al., 2009). In this method, a spinneret connected with a microsyringe pump and the drug–polymer solution is placed into it. The high voltage current (5–30 kV) was supplied to the needle tip to release the charge on the solution surface (Hur & Kim, 2006). A fixed electrical potential is also applied across a fixed distance between the spinneret and the collector (Vo et al., 2013). The electric field accelerates the jar and the used solvent evaporates very quickly to form the micron or submicron diameter fibers. Finally, the sample was collected on the spinning mandrel or screen. The nanosizing and amorphization of the drug incorporated in these fibers lead to enhanced dissolution (Kawakami, 2012). The application of this method has been used to prepare griseofulvin amorphous SD using PVP as a carrier and found stable for 8 months (Srinarong et al., 2009). Yu et al. prepared the SDs using acetaminophen and PVP as the drug and carrier, respectively. The SDs were prepared using electrostatic spinning technique and the comparison was done with the SDs prepared using other techniques. The results of the study revealed that the SDs prepared using this technique showed faster drug release profile compared to other techniques such as vacuum drying, freeze-drying, and heat-drying (Yu et al., 2010).

### 3.8. Supercritical anti-solvent (SAS)

The SAS method is considered an environmentally friendly method to prepare SDs because it does not require an organic solvent. In this method, mostly supercritical carbon dioxide (CO_2_) is used as a solubilizing solvent or anti-solvent. There are a number of favorable properties like the low surface tension, high diffusivity, and low viscosity and the pressure can be easily adjusted. It can easily control the solubility of many drugs (Vo et al., 2013). The drug and used carriers first solubilized in the supercritical CO_2_ and sprayed into an expansion vessel at low pressure through a nozzle. The dissolved drug and carrier droplet quickly converted into SD particles of the desired size. In case of CO_2_ used as anti-solvent, the drug and carrier dissolved in an organic solvent and introduced into the nozzle to spray. After the solution sprayed into the vessel, the organic solvent quickly extracted by supercritical CO_2_ leading to the formation of SD particles of the desired size (Won et al., 2005). The application of this method was performed to enhance the dissolution of irbesartan by preparing SD using Poloxamer as a carrier. The drug:carrier (1:1) was used to prepare the sample and the dissolution results revealed 13-fold enhancement in the dissolution rate than pure drug (Adeli, 2016). In another research, apigenin-nanocrystal was prepared by a SAS method to enhance the bioavailability of apigenin. The study showed that the maximum plasma concentration (*C*_max_) and AUC were increased up to 3.6-fold and 3.4-fold, respectively, in comparison to pure drug (Zhang et al., 2013).

### 3.9. HME technique

The novelty of this method is the conversion of a solid mass of mixed particles into a semisolid mass by the intense mixing and heating. This technique is used to prepare tablets, rods, pellets by blending the drug, carrier, and other excipients (Figure 2). The solid samples were simultaneously mixed, heated, melted homogenized, and finally extruded to form the final formulation (Verhoeven et al., 2009). It helps to give the homogenous products with greater efficiency, within short time and without use of solvents (Gajda et al., 2019). Due to the agitation and intense mixing process forced by rotating the screw during the process, it causes particles disaggregation in the molten polymer to lead to the formation of homogenous dispersion (Vo et al., 2013). The HME samples contain drugs, fusible polymer (one or more), and other excipients like plasticizers and modifiers to prepare the final formulation. In case of the miscible carriers and drugs, there may be a greater chance of formation of amorphous SD and lead to enhanced dissolution profile (Onoue et al., 2013; Vishali et al., 2019). Although there are some miscibility problems between drugs and carriers due to application high shear forces leading to high temperature in the extruder, this method has greater application in the pharmaceutical drug delivery system (Saerens et al., 2011). The effect of HME method was evaluated on the extruded cinnarizine and Soluplus formulation. The result of the study showed that humidity and temperature have a similar effect on the physical stability of Tian et al. (2015). The effect of temperature and humidity were assessed on the prepared SDs with the use of Eudragit^®^ E PO as a carrier and felodipine, carbamazepine, celecoxib, and FB as the drugs. The samples stored at high humidity showed high crystallization than the samples stored at high temperature (Yang et al., 2015). The water solubility was evaluated for β-carotene SDs prepared with the emulsifiers. The water solubility was found maximum with the maximum carrier weight due to their amorphous structure (Ishimoto et al., 2019).

**Figure 2.** Schematic working diagram of hot melt extruder.

Recently, nifedipine and efavirenz-loaded amorphous SDs were prepared using HME method. The SD was prepared using the carrier HPMC-AS and assessed for the solubility and stability of prepared SDs. The findings of the study revealed that the amorphous nature of amorphous SDs was unchanged after 3 months of stability testing at 40 °C and 75% RH. The prepared SD showed the high drug content between 98.98 ± 1.24 and 102.68 ± 0.92%, indicated the stability under accelerated condition. The drug release studies were also evaluated after 3 months of storage and depicted similar release behavior as initial samples (Sarabu et al., 2020). Recently, mefenamic acid (MA) SDs were prepared by HME method using Eudragit VR EPO at two concentrations (20% and 25%) as a carrier. The prepared MA-SDs were characterized for different physicochemical properties, taste masking evaluation, and anti-inflammatory activity. The results of the study revealed conversion to amorphous form from the crystalline state in all SDs in comparison with crystalline spectra of pure MA. The *in vivo* study results showed MA-SDs were capable to mask the bitter taste, significant enhancement in oral bioavailability (*p*<.05) and also found highly efficacious than pure MA (Alshehri et al., 2019). In another study, the effect of magnesium oxide (MgO) and PEG was assessed in the presence of Kollidon 12 PF and 17 PF carriers on the release profile of MA.

The SDs were prepared by HME method. The samples were extruded with twin-screw extruder (16-mm Prism EuroLab, Thermo Fisher Scientific, Carlsbad, CA) at different screw speeds and temperature. The dissolution study results revealed an immediate release pattern with about 80% drug release achieved in 45 min study with SDs containing the combination of MgO, PEG, and Kollidon as compared to the pure drug, binary mixture, and physical mixture (Alshehri et al., 2017). In another research, face-cut melt-extruded pellets of carbamazepine were formulated and HME parameters were optimized using Soluplus^®^ as a polymeric carrier. They found that all the optimized formulations showed good hardness and maximum sphericity (Alshetaili et al., 2016). In another study, the same research group prepared and investigated the solubility enhancement of piperine using different polymers (Eudragit^®^ EPO/Kollidon^®^ VA 64 or Soluplus^®^) by formulating SD using HME technology. The prepared samples were further evaluated for drug release, solubility studies, and permeability characteristics. The findings of the study revealed a significant enhancement in piperine % release, and solubility enhancement was more than 160- and 45-fold in water. Furthermore, the permeability studies result revealed the enhancement in piperine absorption of 10% (Ashour et al., 2016). In another study, HME method was employed to enhance the solubility, dissolution, and bioavailability of aripiprazole loaded SD using Kollidon^®^ 12 PF (PVP) and succinic acid (SA). The solid-state characterizations were performed using SEM and DSC and the results demonstrated the transformation of the crystalline state to an amorphous state in the SDs formulations. The prepared formulation enhanced the solubility, release of drug and also significantly enhanced the oral bioavailability (*C*_max_ and AUC) compared to the pure drug (McFall et al., 2019). In another research work, HME technique was used to improve the physicochemical properties of model drug lansoprazole (LNS) to obtain its stable enteric-coated tablets. Kollidon^®^ 12 PF, Lutrol^®^ F 68, and MgO were selected as the carrier, plasticizer, and alkalizer, respectively. Better release of LNS was obtained by HME SDs tablets compared with the crystalline LNS. MHE LNS was also found as physically and chemically stable after 12 months of storage (Alsulays et al., 2017). Gajda et al. (2018) prepared FFA and nicotinamide loaded cocrystal formulation of via matrix assisted cocrystallization using HME technique (Gajda et al., 2018). They used five different polymers (poloxamer 407, Soluplus^®^, HPMCAS, PVPVA64, PEG-PVA copolymer) to evaluate the physicochemical property of the developed formulation. The prepared formulation showed formation of amorphous composites at different polymer content. There was a significant increase in dissolution was observed for both the used drugs. The ternary SD of carbamazepine: nicotinamide was prepared by extrusion method using the carrier HPMC, SOL, and PVPVA64 (Liu et al., 2012). The formulation was prepared to prevent the thermal degradation of carbamazepine. The ternary SD was prepared in the absence of crystalline phase derived from cocrystal. In another study, tamoxifen (TAM) with resveratrol (RES) loaded ternary amorphous SDs were prepared for breast cancer using the Soluplus, CremophorRH40, and Poloxamer188 as carrier (Chowdhury et al., 2018). The prepared sample showed enhanced dissolution than the drug suspension. The pharmacokinetic study result revealed significant enhancement in drug absorption. The *in vitro* cytotoxicity study was evaluated on MCF7 cells and result showed significantly lesser IC50 value than pure drugs.

### 3.10. Meltrex™

The HME principle is involved in this technique to prepare SD. This is a patented technique and useful for a thermolabile drugs. There are two independent hoppers attached with a special screw extruder to conveying the extruded mass continuously to the extrusion channel. It works very quickly and requires lesser residence time (approximately 2 min) for the material and also avoids the thermal stress to the carrier and drug (Vasconcelos et al., 2007). The temperature during the formulation can be easily regulated between the low temperature of 30 °C to a high temperature of 250 °C (Vo et al., 2013). The drug which is sensitive to oxidation and hydrolysis can be easily prepared because in this process oxygen and moisture are eliminated during the process.

### 3.11. Melt agglomeration

This technique works with high shear mixers or rotary processors. The molten drug and carrier are heated to above the melting point of the binder and sprayed onto the heated binder (van Drooge et al., 2005; Vilhelmsen et al., 2005; Kaur et al., 2012). This process is widely applicable because the temperature can be easily regulated and also high binder content can be added to the agglomerates (Vilhelmsen et al., 2005). The SD of tadalafil was prepared by melt agglomeration technique using Pluronic as a carrier. The pluronics of different grades were melted at 70 ± 2 °C, and then a drug sample was added to the molten carrier. The sample was stirred until a homogenous dispersion was formed. The characterization results revealed uniform dispersion of tadalafil in the carrier matrix. The drug was not completely transformed into the amorphous state but the dissolution rate of tadalafil in Pluronic F-127-based SD was significantly increased compared to the physical mixture (Mehanna et al., 2010). The melt agglomeration method was also used to prepare diazepam SD in a high shear mixing using Gelucire 50/13 and PEG 3000. The prepared SD showed enhanced dissolution at low drug concentration. It showed the high degree of molecular dispersion at the lower concentration (Seo et al., 2003).

### 3.12. KinetiSol^®^ dispersing (KSD) technique

In this process, high energy mixing is performed to get amorphous SDs. It uses a series of rapidly rotating blades to mix the drug and carrier with a combination of kinetic and thermal energy without the aid of external heating sources (DiNunzio et al., 2010). The application of this method employed to prepare itraconazole SD using hypromellose as a carrier. The results of the study revealed that amorphous API was formed within 15 s by KSD technique while HME required over 300 s. The dissolution profile was also improved for the sample prepared by KSD technique compared to the HME process (DiNunzio et al., 2010). The high-resolution atomic force microscopy was utilized to investigate the SDs structure, properties and the interactions between the API and carrier at the molecular level. Yu et al. reported the structure of LNS SD using PVP as a carrier (Yu et al., 2011). There are many conventional and novel SDs preparation techniques reported in the literature. But the selection of appropriate technique depends on the SDs composition and process parameter is crucial to meet the desired goals (Vasconcelos et al., 2016). In case of solvent evaporation method, the organic solvent property is the main factor to check the solubility of drug and carrier. Spray drying and melt extrusion technique have the greater advantage in manufacturing process due to their ability to higher scale up (Vasconcelos et al., 2016).

## 4. Selection of polymer

The selection of ideal polymer in the formulation of SDs is a critical step as it may influence the solubility and dissolution (Školáková et al., 2019), the propensity toward supersaturation (Baghel et al., 2016), and the processability of the ASD (Mohammed et al., 2012). The polymer selection is based on trial and error approach by checking the physicochemical property of drug and carrier (Wu et al., 2011). The factors like glass transition temperature, aqueous solubility, molecular weight, as well as hygroscopicity were considered. The molecular weight of carrier plays an important role in prevention of recrystallization. As the molecular weight increases, the glass transition temperature of the polymer increases and leads to form SDs (if mixed with the API at the molecular level). It will help to increase the stability of SDs during storage by increasing the glass transition temperature. The increase in molecular weight of PVP has shown the reduction of nucleation and crystal growth of piroxicam (Hilton & Summers, 1986). The high molecular weight polymer may give slow drug release from the SDs due to high viscosity of the diffusion layer (Browne et al., 2020).

## 5. Therapeutic efficacy of SDs

There are many pieces of literature that reported the feasibility of SDs as an oral delivery system. The results have reported enhanced pharmacokinetic and pharmacodynamic activities in an animal model. It indicates that SDs are an appropriate technique to improve drug absorption and therapeutic efficacy. Colombo et al prepared Kaempferol loaded SDs and evaluated for antioxidant, anti-inflammatory, and anti-cancer activities. They used Poloxamer 407 as a carrier at 1:5 weight ratio to prepare SDs by the solvent method and melting method. There was 4000-fold enhanced solubility than the free drug. The pharmacokinetic profile after oral administration revealed the AUC and *C*_max_ from SDs were twofold greater than free drug (*p*< .05) in a rat model (Colombo et al., 2019). In another study, ambrisentan loaded SDs were prepared and evaluated for *in vitro* and *in vivo* parameters. The *in vitro* release and *in vivo* bioavailability studies revealed enhanced drug release and drug absorption from prepared SDs after oral administration (Deshmane et al., 2018). Tectorigenin loaded SDs were prepared by a solvent evaporation method using polyvinylpyrrolidone (PVP) and PEG4000 as a carrier in a weight ratio (Shuai et al., 2016). The prepared SDs were characterized for *in vitro* dissolution and *in vivo* bioavailability. The prepared sample showed 4.35-fold higher drug release than that of the free drug after 150 min. The absorption study revealed enhanced AUC_0–_*_t_* and *C*_max_ of TG-SD, which were 4.8- and 13.1-fold respectively in rats. These results confirm the efficacy of SDs for the enhancement of oral bioavailability by increasing its aqueous solubility. The application of oral SDs has been explored in another research by Ofokansi et al., using IBU as drug and PEG 8000 as a carrier. The prepared samples were evaluated for physicochemical characterization, drug release, and anti-inflammatory activity using egg albumin induced paw edema method (Ofokansi et al., 2016). The prepared SDs showed particle size in the range of 113.5 ± 2.5 to 252.5 ± 1.9 μm. There was marked enhancement (*p<.05*) in drug release that was observed in comparison to pure drug and physical mixture. The formulation also showed greater anti-inflammatory activity by achieving edema inhibition (up to 90%) in 6 h, whereas pure drug depicted lesser edema inhibition (77%) in the same time. In another research, ultrafine grinding technology and HME technique were employed to prepare *Angelica gigas* Nakai solid dispersion (AGN-SD) and evaluated for the antioxidant and anti-inflammatory activities (Jiang et al., 2020). From the above findings, the authors concluded that AGN-SDs significantly enhanced biological activities. Luo et al. prepared tanshinone IIA loaded SD to enhance the dissolution, bioavailability, and pharmacological activities (Luo et al., 2020). SDs were prepared via one-pot approach and evaluated for physicochemical evaluation. The prepared SDs showed enhanced dissolution and *in vivo* bioavailability. The sample also revealed enhanced pharmacological activity by incorporating the hydrophobic drug into hydrophilic bio-macromolecules for increasing the release and bioavailability. Apigenin loaded oral SDs were prepared by spray drying method to evaluate the *in vivo* bioavailability on an animal model (Altamimi et al., 2018). The bioavailability of spray-dried apigenin SDs was compared with the marketed and pure apigenin samples. The prepared SDs showed fivefold high *C*_max_ value. The dissolution and bioavailability enhancement was found to be significant with the prepared SDs. The same research group prepared the SD of apigenin using a different method and reported enhanced bioavailability (Alshehri et al., 2019). The pharmacokinetic profile revealed a significant enhancement in oral absorption of apigenin SD prepared using melt technique and microwave technique. The oral bioavailability was enhanced 3.19-fold as compared to a marketed capsule. In another study, the *in vivo* absorption of MA loaded SDs was assessed after oral administration (Alshehri et al., 2019). The samples were further assessed for palatability study and pharmacodynamics study. The optimized mefenamic SD showed enhanced rat palatability and anti-inflammatory activity than pure and marketed formulation. The *in vivo* absorption study result revealed a statistically significant enhancement pharmacokinetic profile than pure MA. The findings of this study suggested that MA SD prepared by hot-melt extrusion method can enhance the therapeutic efficacy after oral administration. The feasibility of aripiprazole loaded SD was evaluated after oral administration by McFall et al. (2019). The prepared aripiprazole SDs showed a marked enhancement in the oral bioavailability (*C*_max_ and AUC_0–12_) as compared to pure drug. In another study, valsartan loaded SD was prepared by using Soluplus^®^ and d-alpha-tocopherol PEG 1000 succinate as a carrier (Lee et al., 2015). The prepared samples were evaluated for a pharmacokinetic profile in rats compared to the oral absorption with the pure drug. The result of the study revealed a significant enhancement in oral absorption than the pure drug. The oral bioavailability of indomethacin loaded SDs prepared with Gelucire 50/13 and Gelucire 48/16 as the carrier was evaluated in a rat model. The samples were prepared by spray congealing method and evaluated dissolution and bioavailability study. The optimized formulation showed considerable enhancement in dissolution (31-fold) and bioavailability (2.5-fold). The application of SDs has been evaluated on another study using andrographolide as drug and HPMC as carrier (McFall et al., 2019). The drug absorption study results revealed a significant (*p*< .05) enhancement in bioavailability compared to pure coarse powder. Rashid et al., (2015) prepared and evaluated ezetimibe loaded solid self nano-emulsifying drug delivery system (SNEDDS), surface modified solid dispersion (SMSD), and the solvent evaporated solid dispersion (SESD) compared to the oral bioavailability with the drug powder (Rashid et al., 2015). All the prepared formulations significantly enhanced the aqueous solubility, dissolution as well as a greater plasma concentration than pure drug. The plasma profile depicted a higher area under the curve in SESD than SNEDDS and SMSD suggesting improved oral bioavailability. In another study, the same research group prepared revaprazan loaded SDs to enhance solubility and oral bioavailability (Park et al., 2019). They used HPMC and Cremophor 25 as carrier and surfactant. The pharmacokinetic profile of prepared SD was evaluated and compared with pure revaprazan powder. The formulation revaprazan/HPMC/Cremophor A25 has the composition (1:0.28:1.12 weight ratio) depicted enhanced drug solubility (∼6000-fold). There was high AUC, *C*_max_, and bioavailability (5.3-fold enhancement) with a faster *T*_max_ value achieved with the prepared SD in comparison to revaprazan powder. In another research, the same research group prepared ezetimibe SDs using HEC and Tween 80 to evaluate the oral bioavailability (Rashid et al., 2015). The ezetimibe loaded SDs showed a marked enhancement in oral bioavailability as compared to pure drug. These studies revealed that SD of poorly soluble drugs after oral administration as an effective technique to enhance the *in vivo* pharmacokinetic and pharmacodynamic efficacy by increasing the solubility and dissolution.

## 6. Mechanism of drug release from SDs

Two main mechanisms are involved in the release of drug from the SDs. In case of the first mechanism, the drug release followed (a) drug controlled release and in second type the release followed (b) carrier controlled release. The prepared drug carrier matrix dissolves or absorbs water quickly due to their hydrophilic property. In some cases, there is a formation of concentrated carrier layer or gel layer. When the drug dissolves in this gel matrix and due to the high viscosity the diffusion of drug diffusion is difficult. It is a rate-limiting step and diffusion of the carrier into the bulk phase. The insoluble or sparingly soluble drug releases into the concentrated layer and release intact after coming in contact with the dissolution media. The release profile also depends upon the particle size, drug solubility, and drug polymorphic state (Craig, 2002). If the drug is partially soluble or entrapped in a concentrated layer then both these two mechanisms work simultaneously. However, these mechanisms help to explain the different release behaviors of SDs and figure out the way to improve the dissolution profile of SDs. These two drugs release mechanism can occur simultaneously because the drug may be partly soluble or entrapped in the concentrated carrier layer. There are several researches that reported the enhancement of drug release as the ratio of carriers in SDs was increased (Srinarong et al., 2009; Alshehri et al., 2017, 2019, 2020; Lavra et al., 2017; Imam et al., 2020). The better drug dispersion in the carrier was achieved with lesser drug crystallinity, and mainly followed drug-controlled release mechanism.

## 7. Patents on SD

Researchers are showing their interest in new methods to enhance the solubility and dissolution rate of poorly water-soluble drugs. Several patents are being filed every year related to the SDs. In this review, we tried to tabulate the published patents on SD, their patent number, publication title, inventor/assignee, and year of publication. The literature review was done from the year 2015 to 2019. Google patents were exploited to search published patent contents. For extensive search, the keywords namely SD was used and the search was filtered to compress the results to last 5 years only. Table 5 tabulates patent number, exact publication title, inventor/assignee, and year of publication of the patent related to SD. In patent US10350174B2 assigned to UCB Pharma GmbH, LTS Lohmann Therapie-Systeme GmbH and Co. KG have talked about SD comprising of a dispersing agent and a dispersed phase. PVP was added for stabilization. It was concluded that the developed system was found to be stable (Wolf et al., 2019). The patent US10231929B2 assigned to Takeda Pharmaceutical Co. Ltd. had achieved improved solubility and absorbability of amorphous pharmaceutical ingredient with one or more substance among methylcellulose and organic acids and an enteric base (Nomura et al., 2019). In patent US20190183852A1 assigned to Kao Corp., nobiletin composition with high water solubility was mixed with hesperidin derivative to develop SD. In this patent, a nobiletin containing composition was produced (Iwashita et al., 2019). In patent US10391103B2 assigned to Sinotherapeutics Inc., ferroporphyrin SD was developed with a carrier in the ratio of 1:1 to 1:10. It was reported to mask the undesirable taste of ferroporphyrin and meliorates irritation with improved bioavailability (Fang et al., 2019). In patent US10265270B2 assigned to Bluelight Pharmatech Co. Ltd., SD of decoquinate was developed by hot-melt extrusion method with a polymeric carrier and 0–10% surfactant. The developed formulation showed improved solubility and better rate of drug release and improved bioavailability (Wang et al., 2019). In patent US10206874B2 assigned to Hetero Res. Foundation, the SD of rufinamide in combination with HPMC as a pharmaceutically acceptable carrier, process for its preparation and pharmaceutical compositions was discussed (Reddy et al., 2019). In patent US10206880B2 assigned to Sandoz AG., the SD of suvorexant with a polymer or a silicon-based inorganic adsorbent was developed as a method for enhancing the quality of sleep in mammals with a sleep disorder as well as a method for controlling obesity (Adamer et al., 2019). In patent US20190269619A1 assigned to Cyclerion Therapeutics Inc., the SD of SGC stimulator was developed with a pharmaceutically acceptable salt for oral consumption (Dunbar et al., 2019). In patent US20190321304A1 assigned to Sunshine Lake Pharma Co. Ltd., lurasidone SD was developed by melting treatment. The developed formulation was reported to have a high dissolution rate and better bioavailability and patient compliance (Xu et al., 2019). In patent US10213433B2 assigned to AbbVie Inc., the SD of a pro-apoptotic agent was developed with a pharmaceutically acceptable polymer carrier and surfactant for oral administration in the management of different types of cancer (Catron et al., 2019). In patent US10322126B2 assigned to Bend Research Inc., the SD of low water-soluble active with an anionic counterion was developed which was reported to have improved bioavailability and dissolution rates (Miller & Morgen, 2019). In patent US20180214422A1 assigned to Veloxis Pharmaceuticals AS., the SD of tacrolimus in a lyophilic vehicle was developed with improved bioavailability (Holm, 2018). In patent US9107830B2 assigned to AbbVie Inc., the SD of an active pharmaceutical ingredient was developed in PEG as water-soluble carrier and PVP or HPMC as crystallization inhibitor was developed (Fort et al., 2015). In patent US9084730B2 assigned to Sanofi SA., the SD of an active pharmaceutical ingredient and pharmaceutically acceptable polymer matrix of polydextrose was developed with improved bioavailability upon oral administration (Bedos et al., 2015). In patent US20150028503A1 assigned to Bend Research Inc., the SD of drugs with concentration enhancing polymers was developed by improved spray drying method by incorporation of pressure nozzle and diffuser plate (Beyerinck et al., 2015). In patent US20150024054A1 assigned to Bend Research Inc., the SD with enhanced bioavailability by spray-dried technique was developed with sparingly soluble drug and hydroxypropyl methylcellulose acetate succinate (Curatolo et al., 2015). In patent US9211261B2 assigned to Bend Research Inc., the SD with immediate release dosage forms by incorporating disintegrant and a porosigen was developed with excellent strength and solubility (Appel et al., 2015).

**Table 5.** List of patent number, publication title, inventor/assignee, and year of publication of patents on solid dispersion system.

Patent no.	Publication title	Inventor/assignee	Reference
US10350174B2	Polyvinylpyrrolidone for the stabilization of a solid dispersion of the non-crystalline form of rotigotine	Hans-Michael Wolf, Christoph Arth, Luc Quere, Walter Müller	Mehanna et al. (2010)
US10231929B2	Solid dispersion	Yukihiro Nomura, Yuki Tsushima, Yutaka Ebisawa	Nomura et al. (2019)
US20190183852A1	Method for producing nobiletin-containing solid dispersion	Masazumi Iwashita, Masahiro Umehara, Shintaro Onishi, Masaki Yamamoto, Keisuke Yamagami, Takaaki Ishigami	Iwashita et al. (2019)
US10391103B2	Ferroporphyrin solid dispersion and preparation method thereof	Larry Yun Fang, Jiansheng Wan, Kun Li, Maojian Gu	Fang et al. (2019)
US10265270B2	Solid dispersion of decoquinate, a preparation process and its application	Hongxing Wang, Yinzhou Fan, Xueqing Chen, Xiaoping Chen	Wang et al. (2019)
US10206874B2	Rufinamide solid dispersion	Bandi Parthasaradhi Reddy, Kura Rathnakar Reddy, Dasari Muralidhara Reddy, Kesireddy Subash Chander Reddy, Bandi Vamsi Krishna	Reddy et al. (2019)
US10206880B2	Solid dispersion comprising an orexin receptor antagonist	Verena Adamer, Andreas Krekeler, Michael Sedlmayr	Adamer et al. (2019)
US20190269619A1	Solid dispersions comprising a sgc stimulator	Craig Anthony Dunbar, Vasu Sethuraman, Ahmad Hashash	Dunbar et al. (2019)
US20190321304A1	Lurasidone solid dispersion and preparation method thereof	Yuzhen Xu, Ning Tian, Xin Huang, Jinsong You, Fangfang Huang	Xu et al. (2019)
US10213433B2	Solid dispersions containing an apoptosis-inducing agent	Nathaniel Catron, David Lindley, Jonathan M. Miller, Eric A. Schmitt, Ping Tong	Catron et al. (2019)
US10322126B2	Solid dispersions of low-water solubility actives	Warren K. Miller, Michael M. Morgen	Miller & Morgen (2019)
US20180214422A1	Solid dispersions comprising tacrolimus	Per Holm	Holm (2018)
US9107830B2	Inhibitors of crystallization in a solid dispersion	James J. Fort, Steven L. Krill, Devalina Law, Yihong Qiu, Eric A. Schmitt	Fort et al. (2015)
US9084730B2	Pharmaceutical composition comprising a solid dispersion with a polymer matrix containing a continuous polydextrose phase and a continuous phase of a polymer other than polydextrose	Michel Bedos, Thierry Breul, Stephen Byard, Isabel Ribeiro Dos Santos	Bedos et al. (2015)
US20150028503A1	Method for making homogeneous spray-dried solid amorphous drug dispersions utilizing modified spray-drying apparatus	Ronald A. Beyerinck, Heather L. M. Deibele, Dan E. Dobry, Roderick J. Ray, Dana M. Settell, Ken R. Spence	Beyerinck et al. (2015)
US20150024054A1	Solid pharmaceutical dispersions with enhanced bioavailability	William J. Curatolo, Scott M. Herbig, James A. S. Nightingale	Curatolo et al. (2015)
US9211261B2	Immediate release dosage forms containing solid drug dispersions	Leah E. Appel, John E. Byers, Marshall D. Crew, Dwayne T. Friesen, Bruno C. Hancock, Stephen J. Schadtle	Appel et al. (2015)

## 8. Future perspectives and strategies

Formulation scientists have shown their interest in drug candidates which are poorly soluble and thus are difficult to be molded into a novel drug delivery system. In the recent times, the application of new carriers, development of novel preparation and characterization techniques and addition of new additives like surfactants, super-disintegrants, and pH modifiers have new hope for the development of more SD products in the future. The novel carries like Soluplus^®^, Kollicoat^®^ IR or Inutec SP1, Inulin^®^, Gelucire^®^, and Pluronic^®^ are used alone or in combination with the different polymers have broadened their application in the formulation of SDs (Tran et al., 2019). Many other novel additives like super-disintegrants, surfactants, and pH modifiers are also exploited these days for enhancing solubility and stability of the active pharmaceutical ingredient (Phuong et al., 2011; Tran et al., 2013). The study by Szuts et al. (2011) exploited sucrose laurate into gemfibrozil-PEG 6000 SDs. The researchers concluded that the dissolution of gemfibrozil in the SD was markedly improved (Szuts et al., 2011). Since, most of the poorly water-soluble drugs have pH-dependent solubility, incorporating pH-modifiers to improve a solubility is a key approach. In a study by Tran et al., the addition of alkalizers in PEG 6000 based system improved the solubility of telmisartan in the SD by modulating the micro-environmental pH and the changing the drug crystallinity (Tran et al., 2008). In another approach by Srinarong et al., (2009), the use of super-disintegrants in SD was found to enhance the dissolution rate by preventing drug crystallization. High energy KSD process is a novel production technique for SDs. They provide the advantage of enhanced mixing, better homogeneity, and reduced processing times over conventional dispersion methods (Srinarong et al., 2009). The prepared SD system by Dinunzio et al. (2010) with KSD process showed improved dissolution rates (Dinunzio et al., 2010). Novel characterization techniques like high-performance DSC, chip calorimetry, nano and localized thermal analysis, high-resolution atomic force microscopy have been introduced which provides better investigational results and eventually helps in overcoming formulation difficulties of SD system. With each progressive approach, we believe that the SD systems will continue to be exploited for formulating poorly soluble drugs.

## 9. Conclusions

SDs strategies have been studied extensively for the enhancement of solubility, dissolution, and bioavailability of poorly water-soluble drugs. To enhance the dissolution and bioavailability of such drugs, the modification of their physicochemical properties is essential. Several natural, synthetic and semi-synthetic polymeric carriers, and surfactant have been studied to modify the physicochemical properties. The reported *in vitro* and *in vivo* (preclinical) investigations have proved the feasibility of SD as a potential carrier for oral drug delivery applications. There are various novel technologies that have been used in the preparation SDs to enhance the biological profile. Nevertheless, clinical studies have been poorly reported on SD systems and hence more *in vivo* studies are also required to support the *in vitro* data.
